The article "Melatonin alleviates myosin light chain kinase expression and activity via the mitogen-activated protein kinase pathway during atherosclerosis in rabbits" was published in 2014. Journal: Mol Med Rep.

# Melatonin alleviates myosin light chain kinase expression and activity via the mitogen-activated protein kinase pathway during atherosclerosis in rabbits

**DOI:** 10.3892/mmr.2014.2753

**Published:** 2014-10-23

**Authors:** XIAOWEN CHENG, YUFENG WAN, YUANHONG XU, QING ZHOU, YUAN WANG, HUAQING ZHU

**Affiliations:** 1 Laboratory of Molecular Biology and Department of Biochemistry, Anhui Medical University, Hefei, Anhui 230032, P.R. China; 2 Department of Clinical Laboratory, The First Affiliated Hospital of Anhui Medical University, Hefei, Anhui 230032, P.R. China; 3 Department of Otolaryngology, The Affiliated Chaohu Hospital of Anhui Medical University, Hefei, Anhui 230032, P.R. China

**Keywords:** melatonin, permeability, myosin light chain kinase, atherosclerosis, mitogen-activated protein kinase

## Abstract

Melatonin (MLT) is an endogenous indole compound with numerous biological activities that has been associated with atherosclerosis (AS). In the present study, rabbits were used as an AS model in order to investigate whether MLT affects endothelial cell permeability, myosin light chain kinase (MLCK) activity and MLCK expression via the mitogen-activated protein kinase (MAPK) pathway. Expression and activity of MLCK were measured using western blot analysis, quantitative polymerase chain reaction, immunohistochemistry and γ-^32^P-adenosine triphosphate incorporation. Endothelial permeability was detected using rhodamine phalloidin fluorescence staining. The phosphorylation of extracellular regulated protein kinase (ERK), c-Jun N-terminal kinase (JNK) and p38 in endothelial cells were also analyzed using western blot analysis. Atheromatous plaques were formed in rabbits with a high cholesterol diet; however, following treatment with MLT, the number and areas of atheromatous plaques were significantly reduced. In addition, MLT treatment reversed the increase of MLCK activity and expression that occurred in rabbits with high cholesterol intake. Furthermore, levels of phosphorylated ERK, JNK and p38 decreased following MLT treatment. In conclusion, the results of the present study indicated that AS may be associated with increased MLCK expression and activity, which was reduced following treatment with MLT. The mechanism of action of MLT was thought to proceed via modulating MAPK pathway signal transduction; however, further studies are required in order to fully elucidate the exact regulatory mechanisms involved.

## Introduction

Atherosclerosis (AS) is a key component of cardiovascular and cerebrovascular diseases, it is one of the most prevalent and severe diseases in the world resulting in high rates of mortality. The pathological mechanism of AS is complex (1). The widely accepted damage-reaction hypothesis postulates that AS is initiated due to endothelial damage (2–4). Endothelial barrier function regulation is known to be associated with cellular signal transduction mechanisms and previous studies have demonstrated that endothelial cell (EC) signal transduction was initiated by increased concentrations of Ca^2+^ (5,6). G proteins activate phospholipase C (PLC), which stimulates the release of Ca^2+^, which further activates protein kinase C (PKC) and myosin light chain kinase (MLCK). MLKC phospharylates MLC, which leads to the rearrangement of EC F-actin and results in increased EC permeability (7–9). The quantity of phosphorylated (p)MLC produced depends on MLCK activity; increased MLCK activity stimulates the contraction of ECs, enlarging the intracellular space, allowing for the infiltration of lipids into the subendothelial layer and therefore accelerating AS pathogenesis (10).

The article "Melatonin alleviates myosin light chain kinase expression and activity via the mitogen-activated protein kinase pathway during atherosclerosis in rabbits" was published in 2014. Journal: Mol Med Rep.

Previous studies have demonstrated that activation of MLCK by extracellular regulated protein kinases (ERK) was crucial for cell migration, which was accelerated by growth factors and integrins (11). Hu *et al* (12) demonstrated that advanced glycation end product (AGE)-induced autophagy via ERK signaling pathways contributed to vascular smooth muscle cell (VSMC) proliferation, which was associated with atherosclerosis in diabetes. Another study indicated that superoxide anion-mitogen-activated protein kinase kinase (MEK)-ERK-MLCK-MLC signaling mediated indoxyl sulfate-induced junctional dispersal of bovine pulmonary artery endothelial cells (13).

Melatonin (MLT) is an endogeneous indole compound associated with numerous biological activities, including circadian rhythm regulation, seasonal changes, sleep, reproduction and cardiovascular functions (14,15). MLT was reported to have marked dose-dependent anti-oxidative effects, acting as a free radical scavenger (16,17). AS is an important disease process associated with the effect of free radicals and chronic inflammatory processes (18,19). Based on the data available, MLT was suggested to have cardioprotective properties via its direct free radical scavenger activity and indirect antioxidant activity (18,20). MLT was reported to contribute to the amelioration of the early phases of AS, including monocyte rolling and invasion of the subendothelial space as well as inhibition of cyclophilin A expression (21).

Previous studies have demonstrated that expression and activity of MLCK were increased in oxidized low density lipoprotein (ox-LDL)-treated human umbilical vein endothelial cells (HUVECs); however, MLCK expression and activity were decreased following treatment with MLT and the ERK1/2 inhibitor PD98059. This study suggested that ox-LDL-induced MLCK expression and activity were associated with phosphorylation of ERK (22). The aim of the present study was to analyze the effects of MLT on EC permeability as well as the activity and expression of MLCK using rabbit AS models. In addition, the role of the MAPK signaling pathway in the association between MLT and MLCK was investigated in order to provide a novel therapeutic target for the treatment of AS.

The article "Melatonin alleviates myosin light chain kinase expression and activity via the mitogen-activated protein kinase pathway during atherosclerosis in rabbits" was published in 2014. Journal: Mol Med Rep.

## Materials and methods

### Animals and groups

New Zealand male purebred white rabbits (four weeks old, 2.0–2.5 kg) were purchased from the Nanjing Rabbit Breeding Farm (Nanjing, China). Rabbits were housed individually in screen-bottomed plastic cages and kept in a temperature-controlled room (25°C) with a standard 12-h light/dark cycle. All experimental and surgical procedures were approved by the Animal Ethics Committee in accordance with the National Guidelines for animal welfare of Anhui Medical University. Rabbits were randomly distributed into three groups: Group I (n=20) was the normal control group in which rabbits were fed a standard diet, group II (n=20) was the AS model group in which rabbits were fed a high-fat diet (standard diet with 5% lard and 2% cholesterol) for 12 weeks, and group III (n=20) was the MLT treatment group in which rabbits were fed the high-fat diet for 12 weeks. From week nine, rabbits in group III were administered 20 mg/kg MLT daily for four weeks (Institute of Clinical Pharmacology, Anhui Medical University, Anhui, China). At the end of the experiment, after 12 weeks all rabbits were anesthetized with an intravenous injection of 3% pentobarbital (Shanghai Healing Biotechnology Co., Shanghai, China), and aortas were then excised and removed. One part of the aorta was fixed in 4% formalin for further analysis through immunohistochemical (IHC) and hematoxylin and eosin (HE) staining. Another part of the aorta was embedded in optimum cutting temperature compound (OCT) (Solarbio Bioscience and Technology Co., Shanghai, China) to produce frozen sections and the remaining portions of the aortas were stored at −80°C for further use.

### Reagents and antibodies

MLT was provided by the Institute of Clinical Pharmacology, Anhui Medical University (Anhui, China). OCT was purchased from Solarbio Bioscience and Technology Co. and γ-^32^P-adenosine triphosphate (γ-^32^P-ATP) was obtained from Yahui Biomedical Engineering Co. (Beijing, China). The IHC kit (streptavidin-peroxidase 9000) was purchased from Zhongshan Jinqiao Biotechnology Co. (Beijing, China). Anti-MLCK antibody (monoclonal antibody produced in mouse; dilution, 1:1,000) was purchased from Sigma-Aldrich (St. Louis, MO, USA), and other antibodies were from Cell Signaling Technology, Inc. (Beverly, MA, USA). All chemicals used were of the highest purity possible.

The article "Melatonin alleviates myosin light chain kinase expression and activity via the mitogen-activated protein kinase pathway during atherosclerosis in rabbits" was published in 2014. Journal: Mol Med Rep.

### Endothelial permeability analysis

Endothelial permeability was detected using surface biotinylation by sulfosuccinimidyl-6-(biotinamido) Hexanoate (NHS-LC-biotin) (Pierce Chemical Co., Rockford, IL, USA) and XRITC-avidin (Pierce Chemical Co.). Frozen aorta sections were incubated with NHSLC-biotin for 30 min. Slides were washed three times (10 min each) with phosphate-buffered saline (PBS) (Shanghai Healing Biotechnology Co.) and air dried, slides were then blocked with 5% (w/v) non-fat milk at 4°C overnight. After washing three times with blocking buffer, sections were then incubated with TRITC-avidin, diluted 1:500 in blocking buffer. Following removal of excess staining solution, slides were washed three times (10 min each) with PBS and air dried. Aortas were then mounted and endothelial permeability was evaluated. Images were captured using an Olympus Provis AX70 system fluorescence microscope (Olympus, Shinjuku, Tokyo).

### MLCK activity assays

Rabbit aortas were homogenized using lysis buffer [1 mM dithiothreitol; 14.5 mM NaCl; 0.5 mM KCl; 0.5 mM MgSO_4_; 10 mM 4-(2-hydroxyethyl)-1-piperazineethanesulfonic acid; 0.5 mM glucose; 0.1 mM phenylmethylsulfonyl fluoride and 1 mM ethylene glycol tetraacetic acid (Shanghai Healing Biotechnology Co.)] on ice. The homogenate was then subjected to three cycles of freeze-thawing to release MLCK and supernatants were harvested following centrifugation at 21,920 × g for 30 min. MLCK activity was calculated using the rate of γ-^32^P-ATP incorporation into MLC. MLCK supernatant (5 μl) was added to 50 μl reaction buffer [20 mM morpholinepropanesulfonic acid, pH 7.4; 2 mM MgCl_2_; 0.25 mM CaCl_2_; 0.2 μM calmodulin (Shanghai Healing Biotechnology Co.); 2 mM γ-^32^P-ATP; and 5 μM recombinant MLC (Yahui Biomedical Engineering Co.)] which was incubated at 25°C for 20 min. The reaction was terminated by pipetting aliquots (40 μl) onto Whatman filter paper (GE Healthcare, Little Chalfont, UK), allowing the paper to dry naturally, rinsing with 75 mM H_3_PO_4_ (Shanghai Healing Biotechnology Co.) three times and then washing several times (5 min per wash) with 95% (v/v) ethanol (Shanghai Healing Biotechnology Co.). Filter papers were then placed in scintillation fluid and measured using a scintillation counter (Tri-Carb. PerkinElmer, Waltham MA, USA). Samples without a substrate were used as blank controls and all experiments were conducted three times.

### Immunohistochemical (IHC) and hematoxylin and eosin (HE) staining

Slices from rabbit aortas were prepared and analyzed using IHC and HE staining as previously described (23,4).

The article "Melatonin alleviates myosin light chain kinase expression and activity via the mitogen-activated protein kinase pathway during atherosclerosis in rabbits" was published in 2014. Journal: Mol Med Rep.

### Reverse transcription quantitative polymerase chain reaction (RT-qPCR) assays

Total RNA from mouse tissues was extracted using TRIzol^®^ reagent (Invitrogen Life Technologies, Carlsbad, CA, USA) and 1 μg isolated total RNA was converted into complementary DNA (cDNA) using a First-Strand cDNA Synthesis kit (Toyobo Co., Ltd., Osaka, Japan). Power SYBR green master mix (Applied Biosystems, Foster City, CA, USA) was added to cDNA samples, which were then subjected to qPCR using the StepOne^TM^ Real time PCR system (Applied Biosystems). Relative MLCK messenger RNA (mRNA) levels were normalized to β-actin, the reference gene. The following primers were used: MLCK mRNA forward, 5′-GAG AGA CTG GAA ACC GAA GAA G-3′ and reverse, 5′-CAG GTC ACG AAT GGT CTT AGA G-3′; and β-actin forward, 5′-CCC AGC ACC ATG AAG ATC AA-3′ and reverse, 5′-CTG CTT GCT GAT CCA CAT CT-3′.

### Western blot analysis

Aortas were homogenized in 1× SDS lysis buffer containing 50 mM Tris-HCl (pH 6.8), 10% glycerol and 2% SDS (Shanghai Healing Biotechnology Co.). The homogenates were boiled for 10 min and then centrifuged at 16,060 × g for 20 min at room temperature. The total protein concentration of each sample was measured using a MicroBCA^TM^ Protein Assay Reagent kit (Pierce Biotechnology, Inc.). Samples were separated using 10% SDS-PAGE and then transferred to polyvinylidene difluoride membranes (GE Healthcare, Piscataway, NJ, USA). Membranes were blocked using 5% (w/v) bovine serum albumin (Amresco, Solon, OH, USA) for 2 h, followed by a 4°C overnight incubation with primary antibodies. Antibodies were purchased from Cell Signaling Technology, Inc. except anti-MLCK antibody. Anti-p38 and anti-JNK antibodies were polyclonal antibodies produced in rabbit. Anti-pp38, anti-pJNK and anti-β-actin antibodies were monoclonal antibodies produced in mouse. The dilution of anti-p38 and anti-JNK antibodies was 1:1,000. The dilution of anti-pp38 and anti-pJNK antibodies was 1:500. The dilution of anti-β-actin antibody was 1:5,000. Primary antibodies were detected using corresponding horseradish peroxidase-conjugated secondary antibodies (Zhongshan Jinqiao) coupled with enhanced chemiluminescence reagents (Engreen Biosystems, Beijing, China). Three independent experiments were conducted to confirm the reproducibility of the results.

### Statistical analysis

Values are expressed as the mean ± standard deviation. Statistical analyses were conducted using multiple comparisons between groups assuming population variances were equal and with normal distributions. Comparisons between two groups were based on least significant differences. P<0.05 was considered to indicate a statistically significant difference between values.

The article "Melatonin alleviates myosin light chain kinase expression and activity via the mitogen-activated protein kinase pathway during atherosclerosis in rabbits" was published in 2014. Journal: Mol Med Rep.

## Results

### Atheromatous plaques and endothelial permeability are reduced in MLT-treated AS model rabbits

As shown in Fig. 1, MLT treatment attenuated the number and area of atheromatous plaques in the aortic walls of rabbits on high cholesterol rabbits compared to those of the AS model rabbits. In order to further assess the cause of atheromatous plaque formation, endothelial permeability was determined using rhodamine phalloidin fluorescence staining. The results demonstrated that endothelial permeability was markedly increased in the AS group compared with that of the control group; in addition, the hyperpermeability of AS rabbits was reduced following treatment with MLT (Fig. 2).

### MLT treatment attenuated MLCK protein and mRNA expression levels, morphological abnormalities and MLCK activity in AS aortas

MLCK protein and mRNA expression levels were demonstrated to be significantly higher in the AS model group compared with those of the control group; however, the MLT treatment group expressed significantly decreased levels of MLCK protein and mRNA compared to those of the AS group (Fig. 3). HE staining showed that normal aortas had tight junctions between cells and a complete tunica intima; however, damage to the tunica intima and the formation of fibrous caps on the surface of plaques were observed in the AS group. Furthermore, following treatment with MLT, these abnormalities in the AS group were less evident (Fig. 3A). As shown in Fig. 4, MLCK activity was significantly increased in the AS group compared to that of the control group; by contrast, following MLT treatment, MLCK activity was significantly reduced compared to that of the AS group (P<0.05) (Fig. 4).

### MLT treatment decreases levels of MLCK, p-extracellular regulated protein kinase (pERK), pp38 and p-c-Jun N-terminal kinase (pJNK)

Western blot analysis of rabbit aortas revealed that protein expression levels of pERK, pp38 and pJNK were markedly increased in the AS group compared with those of the control group (P<0.05), whereas MLT treatment significantly decreased the levels of these phosphorylated proteins compared with those of the AS group (P<0.05) (Fig. 5). Changes in levels of MLCK, pERK, pp38 and pJNK were all comparable, which therefore indicated that hyper-permeability of the aortic endothelium was associated with the expression and activity of MLCK, which may be attenuated by MLT via the MAPK signaling pathway.

## Discussion

Vascular endothelial cells are the first permeability barrier between vascular tissue and blood, which were reported to be important for maintaining normal biological homeostasis (24). It is widely accepted that endothelial injury in arteries initiates the formation of AS lesions. MLCK is a protein kinase that has been reported to have an important role in the reorganization of the cytoskeleton, leading to the disruption of vascular barrier integrity (25); in addition, the mechanism of MLCK action was reported to proceed via the catalysis of MLC phosphorylation, which may lead to cytoskeletal rearrangements (26). Endothelial cell concentric contraction and gap formation are followed by cytoskeletal changes, which facillitates the infiltration of lipids into the arterial intima and accumulation in arterial walls, ultimately leading to atheromatous plaque formation (27).

The article "Melatonin alleviates myosin light chain kinase expression and activity via the mitogen-activated protein kinase pathway during atherosclerosis in rabbits" was published in 2014. Journal: Mol Med Rep.

The results of the present study demonstrated that MLT anti-AS effects were associated with the expression and activity of MLCK regulated via MAPK phosphorylation. A rabbit model of AS was established through a sustained high-fat diet. Atheromatous plaques were found to be deposited on the arterial walls of these rabbits. The lipid infiltration and endothelial injury hypothesis are widely used to explain the pathogenesis of AS (28). In the present study, Rhodamine phalloidin fluorescence staining demonstrated that endothelial permeability was significantly increased in AS. Permeability was previously reported to be regulated via complex interactions between signaling molecules and structural proteins in the endothelium, including adhesive cell-cell and cell-matrix contacts, which occurred between junctional proteins and focal adhesion complexes in the cytoskeleton (8). At the beginning of the present study it was hypothesized that the change in arterial intima integrity may be associated with increased activity and expression of MLCK. The results of the present study confirmed that MLCK expression and activity were significantly increased in the AS group compared with those of the controls. These results therefore indicated that MLCK activity and expression may have a crucial role in AS.

Previous studies have demonstrated that following ERK pathway suppression, MLCK and downstream pMLC expression levels were decreased in leptomeniges carcinomatosis-MCF-7 cells, indicating that ERK1/2 may regulate MLCK and its phosphorylation (29). In addition, a previous study revealed that the expression and activity of MLCK induced by ox-LDLs were associated with ERK phosphorylation (22). ERK is a member of the MAPK family, which also includes the highly conserved Ser/Thr protein kinase, p38 and JNK. Studies have demonstrated that p38 MAPK had an important role in regulating burn-induced intestinal permeability via the activation of MLCK; in addition, p38 inhibition was reported to be a potential therapeutic target for the attenuation of the breakdown of the intestinal barrier through the prevention of burn-induced modifications of tight junction proteins (30). Phosphorylation cascades were reported to trigger biochemical and conformational changes in the barrier structure of the endothelium, which may lead to the induction of unwanted paracellular pathways (8). The results of the present study demonstrated that phosphorylation levels of ERK, p38 and JNK were markedly increased in the AS group; in addition, the changes in expression of pERK, pp38, pJNK and MLCK were comparable. This therefore indicated the use of protein kinase inhibitors as potential therapeutic agents for the prevention and treatment of endothelial hyperpermeability and vascular barrier dysfunction.

The article "Melatonin alleviates myosin light chain kinase expression and activity via the mitogen-activated protein kinase pathway during atherosclerosis in rabbits" was published in 2014. Journal: Mol Med Rep.

MLT is an endogeneous indole compound, which is synthesized and secreted by the pineal body in vertebrates. Previous studies have shown that MLT had potent antioxidant properties that may prevent the development of AS (31). It has also been reported that the expression and activity of MLCK, induced by ox-LDL, was significantly decreased by MLT. The results of the present study demonstrated that MLT attenuated the formation of atheromatous plaques and reversed the increase of endothelial hyperpermeability as well as MLCK expression and activity in AS model rabbits. This therefore indicated that AS may be associated with MLCK expression and activity, which may be reduced by MLT via the MAPK signal transduction pathway.

In conclusion, the results of the present study provided evidence from animal models that changes to the endothelial cytoskeleton affected endothelial function. MLCK-mediated MLC phosphorylation was suggested to have an important role in the development of AS. MLT served as a switch for modulating the activity and expression of MLCK via the MAPK pathway involving its downstream signaling molecules ERK, p38 and JNK. However, further studies are required to localize components of the pathways and to examine their interactions and mobility in order to elucidate the exact regulatory mechanisms involved in the effect of MAPK cascades on MLCK.

## Figures and Tables

**Figure 1:** A comparison of arterial wall appearance of rabbits from each group. Atheromatous plaques were obvious in the AS group compared to the control. Following treatment with MLT the numbers and areas of atheromatous plaques were reduced compared to those in the AS group. Con, control; AS, atherosclerosis model group; MLT, melatonin-treated AS group.

**Figure 2:** MLT reverses the hyper-permeability of the arterial intima induced by a high-fat diet. Following incubation with NHS-LC-biotin for 30 min, frozen sections were incubated with XRITC-avidin in order to localize surface-bound biotin. NHS-LC-biotin reacts with molecules in the plasma membranes of the endothelial cells of aorta intima, which together appear as a thick, continuous line at the surface of the aorta intima in the normal rabbit. In contrast, we observed the biotin molecules penetrated into subendothelial spaces demonstrating the disruption of the tight junction seal of the aorta intima in AS group and MLT group. However, the hyperpermeability of AS rabbits was reduced following treatment with MLT (magnification, ×20). Con, control; AS, atherosclerosis model group; MLT, melatonin-treated AS group.

The article "Melatonin alleviates myosin light chain kinase expression and activity via the mitogen-activated protein kinase pathway during atherosclerosis in rabbits" was published in 2014. Journal: Mol Med Rep.

**Figure 3:** MLT decreases MLCK protein and mRNA expression. (A) Immunohistochemical analysis using anti-MLCK antibodies to determine the expression of MLCK in the artery wall and HE staining to detect the integrity of arterial intima. (B) Western blot analysis of MLCK proteins in the artery walls. (C) MLCK mRNA expression in artery walls was analyzed by quantitative polymerase chain reaction. ^*^P<0.05 vs. control; ^#^P<0.05 vs. AS group. Each assay was repeated three times. Con, control; AS, atherosclerosis model group; MLT, melatonin-treated AS group; MLCK, myosin light chain kinase; mRNA, messenger RNA; HE, hematoxylin and eosin.

**Figure 4:** MLT decreases MLCK activity in the artery wall. MLCK activity was measured by rates of γ-^32^P-adenosine triphosphate incorporation into MLC as the substrate. ^*^P<0.05 vs. control; ^#^P<0.05 vs. AS group. Each assay was repeated three times. Con, control; AS, atherosclerosis model group; MLT, melatonin-treated AS group; MLCK, myosin light chain kinase.

**Figure 5:** MLT decreases MAPK activation in the artery wall. Western blot analysis of (A) ERK, (B) p38 and (C) JNK activation using phosphospecific antibodies. ^*^P<0.05 vs. control group; ^#^P<0.05 vs. AS group. Each assay was repeated three times. ERK, extracellular regulated protein kinase; JNK, c-Jun N-terminal kinase; p-, phosphorylated; MAPK, mitogen-activated protein kinase; Con, control; AS, atherosclerosis model group; MLT, melatonin-treated AS group.
